# Participation of Soccer Training Improves Lower Limb Coordination and Decreases Motor Lateralization

**DOI:** 10.1155/2022/7525262

**Published:** 2022-04-30

**Authors:** Selcuk Akpinar

**Affiliations:** Faculty of Sport Science, Nevşehir Hacı Bektaş Veli University, Turkey

## Abstract

Athletes, who display less lateralization, are considered to be more successful in their sports. Therefore, it is important to test the lateralization profiles of the athletes to determine future prospects. Soccer is one of the sports where lateralization plays an important role because performing the passes and kicks with either foot may increase the success rate. Improved lower limb coordination is also very essential to perform the soccer skills more efficiently. Thus, the purpose of this study was to investigate the motor lateralization profiles of youth soccer players and to compare the same lateralization to non-athletes. A total of 28 healthy youth (14 soccer players) aged between 14 and 16 years voluntarily participated in this study. All participants were right-footed and were asked to hit the targets with their either foot maintaining accuracy in a custom-made virtual reality interface. Final position error (FPE) and foot path deviation from linearity (FPDL) were calculated to test motor lateralization for each foot and group. Two-way Mixed Model ANOVA was conducted for each dependent variable. Results indicated significant differences for FPDL between groups, while there were no significant differences between groups and within feet for FPE. Nonathletes had significantly higher FPDL with their nondominant foot compared to their dominant foot, which was not observed among soccer players. Overall, nonathletes' movements were more curvature path compared to soccer players, thus, can be considered as less coordinated. As soccer players did not show a difference between their feet on FPDL and performed better than nonathletes, soccer participation can improve lower limb coordination as well as alter motor performance and lateralization.

## 1. Introduction

Soccer is one of the most popular sports in more than 200 countries [1]. Approximately 270 million people (4% of the world population) actively participate in soccer [2, 3]. This popularity may be due to the fact that both gender like watching and playing it in a wide age range, and it does not require any specific physical features and anthropometric parameters at the amateur level. In contrast to the amateur level, playing soccer at expert-level requires highly developed physical capacities, psychological factors, perceptual, cognitive, and motor skills such as running, jumping, heading, kicking, passing, dribbling, and balance [3–5]. All of those capacities are determined player's performance level with (i.e., passing, shooting, heading, controlling, and dribbling) and without the ball (i.e., running, walking, and jumping) in a soccer match [4, 6]. Additionally, technical skill is also known as specific motor skill (i.e., passing, shooting, heading, controlling, and dribbling) and assessed according to kicking performance by measuring some parameters such as kicking accuracy and ball velocity [7, 8]. Further, the ball accuracy and velocity are affected by leg preference [9]. Leg preference or footedness is defined as the tendency to select one leg for various motor functions in opposed to other in performing motor tasks, such as kicking a ball [9, 10]. Previous research focused on the functional advantages of the dominant leg over the nondominant one for accuracy [11], kicking speed [8, 12, 13], reaction time [14], and balance [15]. These findings suggest that each foot was used for different tasks [16]. For example, in the process of kicking or passing, the dominant leg is preferred to perform kicking while the nondominant leg is preferred to provide balance (stabilization) [16]. 79.2% of top-class soccer players in FIFA World Cup 1998 preferred their dominant foot in mobilization skills (i.e., free kick, penalty kick, corner kick, and goal kick) to perform the tasks more accurately and powerfully, while the nondominant foot was preferred only in passing when it is required.

Whereas a human body was created as a symmetric structure, functional movements could be asymmetric between two limbs [16–19]. When there are a 10% or more differences between two limbs in a movement quality (force, power, or muscle girth), it is assumed that motor lateralization exists [11]. Motor lateralization was also related to neural control, explained by a theory called “dynamic dominance of motor lateralization.” According to this theory, the left hemisphere/right arm is specialized for coordination while the right hemisphere/left arm specialized in the stabilization of the movement [19]. This specification may be also valid for the legs as there was a significant association between handedness and footedness dominance [20–22]. As stated above, motor lateralization should play an important role in soccer as the dominant leg performs most of the skills more accurately and powerful than the nondominant one [11]. Even though soccer players display lateralized behaviors when preferring a foot to execute passing or shooting skills, it has been previously shown that less lateralized behaviors are considered to be an efficient factor in order to be a professional soccer player [11, 23–25]. Therefore, one of the common features of top-class soccer players about lateralization is that they have applied extensive soccer-specific training to use both feet very well, and thus, they become less lateralized players [9, 16, 23]. The effect of lateralization on performing movements is important and plays a major role in soccer performance. Especially, the youth period is very important for learning new movement patterns with both feet so that the player could be more successful to perform those skills during the game-like situation [1]. In this regard, it was thought that the lateralization level of the soccer players should be determined in the beginning of the youth period to develop the bilateral competence of each foot for better motor performance [26]. Moreover, it is also important to measure if long-term participation in soccer training may alter motor lateralization. Therefore, the purpose of this study was to investigate motor lateralization profiles between youth soccer players and youth nonathletes.

## 2. Materials and Methods

### 2.1. Participants

A total of 28 healthy male participants aged between 14 and 16 years volunteered in this study. Fourteen participants were soccer players (*M*_age_ = 14.79 ± 0.80 years), and fourteen age-matched (*M*_age_ = 14.93 ± 0.73 years) control participants had no training experience in any sports. Soccer players had 3-5 years of soccer playing experience. Participants were determined as a convenience sampling method and were recruited from the local soccer teams. All participants were right dominant footed, which was determined by kicking a ball [27]. All individuals and their parents signed the consent form approved by the Institutional Review Board of the Nevsehir Haci Bektas Veli University (permit no: 2018.10.110), and the study was conducted according to the declaration of Helsinki as amended by the World Medical Association Declaration of Helsinki.

### 2.2. Experimental Setup and Task

Participants stood on a 20 cm height platform from the ground with either leg parallel to a 55” LCD TV, which is located 2 m away from the participants (Figure 1) and 10 cm above the ground. A sensor of the electromagnetic movement tracker (TrackSTAR, Ascension Technology, USA) was placed on the participants' big toes of the foot being measured. A simultaneous 2D view of the kicking leg was provided to the participants as a visual feedback. A custom-made virtual reality interface provided a cursor representing tip of big toe, a start circle, and 3 different targets on the feedback screen. The cursor represented the tip of the big toe of each foot, and its position on TV was updated in real time, which was 100 Hz.

Three targets (0^0^, 10^0^, and 20^0^ from the start circle) were presented in a randomized order, and the task was to hit these targets with considering accuracy. One target was displayed for each trial. The start circle with a diameter of 3 cm was aligned with the height of the supporting platform and was 30 cm away from the starting position. Targets were displayed as 5 cm in diameter. The cursor was 1.5 cm in diameter with cross hair. There was an audio go signal with visual information upon which participants were asked to move to the target. The participants had to put the cursor inside the start circle for 300 milliseconds to initiate the movement. The task was to move the cursor to each target in 1-sec duration. The initiation of the movement was self-paced, thus, the participants had enough time for the movement planning. Participants performed a total of 20 trials for each target. Thus, each participant made 60 trials with their each foot. For motivational purposes, the accuracy of each trial was rewarded with 10, 3, and 1 point for locating 5 cm, 6 cm, and 7 cm diameter from the center of the displayed target, respectively. The task was performed by each foot, and the foot being tested was counterbalanced among the participants.

### 2.3. Data and Statistical Analysis

To determine motor lateralization, two measures were defined: (1) movement accuracy that was defined as final position error (FPE), and (2) movement quality that was defined as foot path deviation from linearity (FPDL). The FPE was calculated as the Euclidian distance between the last point of the tip of the big toe represented by the cursor and the center of the target. The FPDL was calculated as the ratio between the minor and major axis of the foot path of the big toe. It is considered to be a measurement of coordination. The less values for the FPDL represent more linear movement. Data collection and analysis were performed using custom-made Matlab software.

For statistical purposes, the mean value of each dependent variable was calculated, and analysis was performed for each dependent variable. Two-way mixed model ANOVA was conducted to test if each dependent variable was different within the foot and between the groups using IBM SPSS Statistics (Version 23 for Windows; IBM, Armonk, NY, USA). Thus, foot (dominant and nondominant) was treated as a within-factor, and groups (youth soccer players and nonathletes) were treated as a between-factor. The student's *t*-test with Bonferroni correction was conducted for post hoc analysis. The statistical significance level was set as *p* < 0.05.

## 3. Results

Figure 2 displays the mean value of final position error (FPE) for dominant and nondominant foot and groups (youth soccer players and nonathletes). Overall, both groups displayed similar performance between feet in terms of FPE. A 2-way mixed-model ANOVA with foot as within-factor and groups as between-factor revealed no significant main effects and nor interaction, *F*_(1, 26)_ = 0.61, *p* = 0.87, and *η*^2^ = 0.02 for foot main effect; *F*_(1, 26)_ = 0.07, *p* = 0.93, and *η*^2^ = 0.003 for group main effect; *F*_(1, 26)_ = 0.02, *p* = 0.97, and *η*^2^ = 0.001 for foot x group interaction.

Figure 3 shows the mean value of foot path deviation from linearity (FPDL) for dominant and nondominant foot and groups (youth soccer players and nonathletes). Youth soccer players had similar FPDL performance for dominant and nondominant foot, which was not observed in youth nonathletes. A 2-way mixed model ANOVA displayed a significant foot main effect, *F*_(1, 26)_ = 11.66, *p* < 0.01, and *η*^2^ = 0.31; a significant group main effect, *F*_(1, 26)_ = 4.01, *p* < 0.05, and *η*^2^ = 0.13; and a foot x groups interaction *F*_(1, 26)_ = 9.11, *p* < 0.05, and *η*^2^ = 0.26. The dominant foot's FPDL (*M* = 0.087 ± 0.014) was significantly better than the nondominant foot (*M* = 0.097 ± 0.019). Youth soccer players (*M* = 0.086 ± 0.018) had better FPDL than youth nonathletes (*M* = 0.098 ± 0.016).

*Post hoc* analysis for two-way interaction displayed that in nonathletes, the nondominant foot (*M* = 0.11 ± 0.015) had significantly larger FPDL than the same group's dominant foot (*M* = 0.088 ± 0.011), while they were larger than the values obtained from soccer players' both feet (*M*_Dominant_ = 0.086 ± 0.018 and *M*_Nondominant_ = 0.087 ± 0.019). Moreover, there was no significant difference in FPDL between feet in youth soccer players.

## 4. Discussion

This study investigated motor lateralization profiles of youth soccer players and nonathletes to test if soccer players display a lateralized performance between their feet. Moreover, motor performance of the feet between youth soccer players and youth nonathletes was compared. The results displayed no significant differences between both groups and within feet for the final position error (FPE). That is, the dominant and nondominant feet had similar accuracy performance in both groups. However, a significant difference was found for foot path deviation from linearity (FPDL). Nonathletes' nondominant foot had worse FPDL compared to dominant foot, which was not observed in soccer players. Thus, whereas nonathletes displayed a lateralized pattern in FPDL, soccer players did not have this pattern in FPDL. The reason to have similar FPE between both groups and within feet may be because all participants focused on the task, which included putting the cursor into the target with their each foot. Although both groups focused similarly to kick the target, soccer players focused on the quality of the kick more (better FPDL) than nonathletes with their both feet. Participating sports activities were found to modify motor lateralization of the arms [17, 28]. That is, the less lateralized motor performance of the arms was observed in different types of sports. In fact, although foot motor performance measurements were taken in the current study, similar findings were obtained.

While there are many studies investigating motor lateralization of the arms in different sports [28, 29], only a few studies focused on foot lateralization in sports. Motor lateralization is essential for successful performance in many sports, which include bimanual tasks (e.g., basketball, water polo, soccer, and volleyball). Less lateralized movements can improve technical skills and thus have positive effects on the game situations. When we consider soccer, it is important to be able to use both feet depending on different game positions [24]. In fact, Haaland and Hoff (2003) [23] found an improved bilateral motor performance of soccer players after 8-week nondominant leg training. In this study, a better motor performance of the nondominant foot in FPDL for the soccer players compared to nonathletes was observed, which is in line with the aforementioned findings. FPDL can be considered to require the coordination pattern of the leg. That is, in order to have better FPDL, leg joints should have good and efficient coordination to perform the kicking task applied in the current study. In this essence, participation of the soccer trainings might improve the lower limb coordination pattern besides other physical fitness parameters.

In modern soccer, players should be able to use their either foot for all technical skills. This could improve the performance of the player, which could help to increase the probability of winning the game. For instance, less lateralized attackers fake the defenders by using their either foot and find opportunities to score a goal [24, 30]. Less lateralized defenders, on the other hand, may be able to tackle the ball away from the defensive zone more quickly and effectively than lateralized attackers [19]. Previous studies have shown that soccer players who can use their both feet showed less lateralized foot behaviors, and thus, they are regarded as a desirable skill at the top-class level and have more successful performance than lateralized soccer players [11, 23–25]. One of the common features of top-class soccer players is that they have applied extensive soccer-specific training to use both feet very well and develop their motor performance level [9, 16, 23]. Therefore, it can be suggested that all coaches working with youth should also include nondominant foot practices in the training program to reduce the level of lateralization.

The soccer coaches should be conscious that players use their both feet during the training sessions. In this case, it may be possible for the soccer players to perform soccer-specific technical skills accurately and efficiently with both feet during the game. It is precisely recommended that coaches should motivate and encourage their players to use both feet. Furthermore, more than 50% of the registered soccer players worldwide were youth athletes [31], thus, it is important to improve their foot motor performance and to teach the players to use both feet at younger ages.

## 5. Conclusions

Participation of sports activities has many beneficial effects on physical fitness levels. More specifically soccer training was found to improve weight, height, BMI, and standing long jump among the youth [32]. In the current study, it has been also found that soccer training improves the lower limb coordination and decreases the motor lateralization. It might be beneficial to use foot motor performance measurements for the talent identification in soccer in order to get less lateralized players at the initial stage. In this current study, the soccer players who participated in this study were not selected by their soccer clubs with the measurements of their motor lateralization profiles. Thus, the better performance in lower limb coordination observed in the study might stem from the participation of soccer trainings. Future studies may focus on the longitudinal measurements of the motor lateralization to track the changes throughout the times.

## Figures and Tables

**Figure 1:** Experimental setup.

**Figure 2:** The mean value of final position error (FPE) for dominant (black in color) and nondominant foot (grey in color) and groups (youth soccer players and nonathletes).

**Figure 3:** The mean value of foot path deviation from linearity (FPDL) for dominant (black in color) and nondominant foot (grey in color) and groups (youth soccer players and nonathletes). ∗ represents *p* < 0.05.

## Data Availability

The datasets analyzed during the current study are available from the corresponding author on reasonable request.
